The article "Construction of a Diagnostic Model for Lymph Node Metastasis of the Papillary Thyroid Carcinoma Using Preoperative Ultrasound Features and Imaging Omics" was published in 2022. Journal: J Healthc Eng.

# Construction of a Diagnostic Model for Lymph Node Metastasis of the Papillary Thyroid Carcinoma Using Preoperative Ultrasound Features and Imaging Omics

**DOI:** 10.1155/2022/1872412

**Published:** 2022-02-08

**Authors:** Chao Zhang, Lihua Cheng, Weiwen Zhu, Jian Zhuang, Tong Zhao, Xiaoqin Li, Wenfeng Wang

**Affiliations:** ^1^Department of Ultrasound, The Affiliated Changzhou No. 2 People's Hospital with Nanjing Medical University, Changzhou 213004, China; ^2^Graduate School, Dalian Medical University, Dalian 116000, China; ^3^School of Science, Shanghai Institute of Technology, Shanghai 201418, China

## Abstract

In this paper, we mainly adopted 337 patients who had undergone the surgery on lymph node metastasis of papillary thyroid carcinoma (PTC) as the sample population. In order to provide clinical reference for the intelligent decision-making in treatment plan and improvement of prognosis, we utilized ultrasound features and imaging features to construct five early diagnosis models for patients based on the ultrasound features, imaging features, and combined features. The model integrated with broad learning system (BLS) showed the best performance, with the area under the curve (AUC) of 0.857 (95% confidence interval (CI): 0.811–0.902)) and the accuracy of 0.805 (95% CI: 0.759–0.850). For demographic and clinical features, the prediction effect was also good, with the AUC more than 0.700.

## 1. Introduction

Papillary thyroid carcinoma (PTC) is one of the most common pathologic types of thyroid cancer [1]. The current clinical problem is to find regions where lymph node metastasis is prone to occur [2]. This problem is usually solved by utilizing the ultrasound technology, which is also the first choice for thyroid cancer examination. Ultrasound technology can determine whether the patient has cervical lymph node metastasis before surgery, which is of great significance for the selection of surgical methods, radiotherapy and chemotherapy, and the judgment of prognosis [3]. The major advantage of machine learning is that the learning model can improve treatment decisions for cancers and provide clinical references to improve the prognosis [4]. Deep learning models have been used in previous studies, but it takes a lot of time in training stage [5–7].

As an effective and efficient incremental learning system, broad learning system (BLS) can provide value for prediction model, which largely reduced the time cost of model training [5]. If combined with imaging omics, broad learning features can then be utilized in establishing the lymph node metastasis model [6–8]. Imaging omics is mainly based on the extraction and analysis of images features from CT, MRI, PET, and other medical images to quantitatively evaluate diseases such as thyroid papillary carcinoma and lymph nodes [9]. It can be used to diagnose diseases, predict prognosis, and analyze biological behavior of diseases [10]. Imaging omics was proved to be objective in image extraction of lymph node features in PTC and had important implications for prediction of clinical outcome [11–15]. Since imaging omics has been successfully applied to the diagnosis of thyroid cancer, lung cancer, liver cancer, breast cancer, and other diseases [16–22], it will also be employed in the present study.

To combine imaging omics with broad learning features, random forest is employed to develop the basic analytic models, which is a combination of decision trees [23]. Each decision tree is trained by randomly generating a new data set from the original data set. The result of random forest is the decision of most decision trees [24–28]. But a single model classification method is often prone to overfitting problem. Many scholars often improve the prediction accuracy through the combination of multiple single models, which is called classifier combination method. Random forest is an algorithm that proposed to solve the overfitting problem of a single decision tree model [29]. Random forest uses the bootstrap resampling method to extract multiple samples from the original samples and then conducts decision tree modeling for each bootstrap sample, and then synthesizes multiple decision trees for prediction, and obtains the final prediction result through voting [30, 31].

The organization of this article is as follows. We will use preoperative ultrasound features and image analyses to construct an early diagnosis model for lymph node metastasis in PTC in Section 2. These models will be performed, evaluated, and then integrated with BLS in Section 3.

## 2. Materials and Methods

### 2.1. Study Design and Population

This study was a cross-sectional study which was approved by the Institutional Review Board of The Affiliated Changzhou No. 2 People's Hospital with Nanjing Medical University (approval number: [2021]KY021-01). The sample population was 337 patients who had undergone PTC surgery in Changzhou Second People's Hospital after inclusion and exclusion.

The inclusion criteria were as follows: (1) patients aged ≥18 years old; (2) PTC patients who received fine needle biopsy before operation and were confirmed; (3) patients without benign lesions or single malignant lesions; (4) patients who underwent extensive neck lymph node dissection; (5) patients with complete clinical data.

The exclusion criteria were as follows: (1) patients who received anticancer treatment such as radiotherapy and chemotherapy before operation; (2) patients without undergoing ultrasound examination before operation.

### 2.2. Missing Data Assessment

There were 428 nodules in 337 patients. Noting that each nodule had two or more ultrasound images from different angles, there were a total of 973 ultrasound images for 428 nodules in 337 patients. Alternatively, a total of 428 data and 973 representative ultrasound images were collected. Missing values in the data were filled by random interpolation. Sensitivity analysis before and after gap-filling is shown in Table 1.

### 2.3. Image Preprocessing and Classification

In the present study, Lasso regression filtering is used for image processing [32, 33]. The processes were to sample *n* original sample data with the sample size of N and each observation object had an equal probability of being selected, which was 1/N. The sample was regarded as the whole, and the subsamples sampled were regarded as samples from the sample. Such subsample was called the bootstrap sample. The sampling process can be formulated as follows. Let H(x) represent the random forest classification result, *h*_*i*_(*x*) represent the classification result of a single decision tree, Y represent the classification target, *I*(·)  represent indicative function, and the random forest classification model adopt a simple voting strategy to complete the final classification.

1. Each decision tree was generated by training sample *X* with sample size K and random vector *θ*_*k*_
2. Random vector sequence {*θ*_*k*_,  1,…, *K*} was independently and identically distributed
3. Random forest was the set of all decision trees {*h*(*X*, *θ*_*k*_),  *k*=1,2,…, *K*}

Among these processes, each decision tree model *h*(*X*, *θ*_*k*_) had one vote to select the classification result of input variable X: $H\left(x\right)=\underset{Y}{\max}\sum_{i=1}^{k}I\left(h_{i}\left(x\right)=Y\right)$_._

The remaining variable of image feature was gray-level size zone matrix (GLSZM) entropy. The remaining three variables were gender, age, and carcinoembryonic antigen in the demographic information and clinical data, and the remaining four features were the maximum diameter of nodule in ultrasound features, aspect ratio, calcification, and relative capsule position. BLS was established for image classification through learning the variables in the model to obtain the output variables. In the process of image classification, broad learning mapped the input data, constructed the mapping features, and then activated the mapping features to enhance the features, and output the two parts together. We screened out the new features by using the loss function of the 1-norm in Lasso regression, and the new features were merged into the random forest as follows:

(1) $$\begin{array}{c} J\left(w,b\right)=\frac{1}{2m}\underset{w,b}{\arg\;\min}\sum_{i=1}^{m}{\left({\hat{y}}_{i}-y_{i}\right)}^{2}+\alpha \sum_{i=1}^{n}\left\|w_{i}\right\|. \end{array}$$

### 2.4. Establishment of the Diagnostic Models

For each nodule, the ROI was delineated according to the gray image selected in the largest long axis cross section. The early diagnosis model of lymph node metastases (LNM) was constructed by combining the preoperative ultrasound features and ultrasound image features, as shown in Figures 1(a) and 1(b). The focus area of PTC was framed by the clinician, and then the imaging features of the focus area were extracted by the pyradiomics algorithm.

The strategy in construction of the five diagnostic models was different. In Model 1, only demographic information and clinical data were used. In Model 2, we combined demographic information, clinical data, and ultrasound features. Model 3 combined demographic information, clinical data, and imaging features. Model 4 combined the demographic information, clinical data, ultrasound features, and imaging features. Broad learning was used to learn the variables in Model 4, and new variables were obtained, which were incorporated into the random forest model to obtain Model 5.

The data set was randomly divided into 7 : 3 training set and testing set, which were then normalized, respectively. Lasso regression was used to filter features in the training set, and then the prediction model was constructed.

The area under the curve (AUC), accuracy, sensitivity, and specificity were used to evaluate the model. Then, the importance of features was expressed by using the feature importance map.

## 3. Results and Discussion

### 3.1. Diagnostic Performance of the Five Models

As shown in Table 2, because the data were randomly divided into training sets and testing sets, the ultrasonic features were compared in balance. Because their *P* values were all >0.05, the difference between training sets and testing sets was not statistically significant. This confirmed that the performances between training sets and testing sets were comparable.

As shown in Table 3, it can be found from the prediction results that Model 4 performed best in the testing set, which combined ultrasound features and imaging features in our data set, with the AUC of 0.857 (95% confidence internal (CI): 0.811–0.902) and the accuracy of 0.805 (95%CI: 0.759–0.850). The receiver operator characteristic (ROC) curves of the four models are shown in Figure 2.

### 3.2. Prediction Results after Integrated with Broad Learning

Eight features in Model 4 were included in BLS model to get 106 features, and then 5 features were screened out by Lasso using *α* = 0.004. Five features put into the stochastic forest prediction model to predict whether lymph node metastasis occurred are shown in Table 4.  Figure 3 shows the ROC curve of Model 4 and Model 5 in training and testing sets.

### 3.3. Discussion on the Importance of Model Features

Since the prediction results of Model 4 and Model 5 were relatively close, and the difference was not statistically significant, we finally chose Model 4 because of its high interpretability. From the map of feature importance (Figure 4), it can be found that the most important variable was the maximum diameter of nodules, followed by GLSZM zone entropy in imaging features, and the third was carcinoembryonic antigen.

Overall, carcinoembryonic antigen and age were the best predictors of demographic and clinical features. Among ultrasonic features, the maximum diameter of the nodule was the best predictor. Imaging features also predict well, as seen in Figure 5.

As the most common thyroid malignancy, the papillary thyroid cancer is associated with cervical lymph node metastases in 30% to 90% of patients [34]. The lymph node dissection (LND) is the mainstay treatment for clinically evident cervical lymph node metastases [35]. So far, surgical treatment options in the literature include the traditional radical LND, the modified radical LND, the selective LND, and a “berry picking” resection in which only the grossly abnormal lymph nodes are excised [36–42]. The selective LND represents a compartment-based resection based on documented lymph node metastases [43, 44]. This study constructed diagnostic models through an integration of the random forest and BLS, which was demonstrated to be a successful attempt to break the related bottlenecks in the future.

Before constructing the diagnostic models for lymph node metastasis, we considered using the ultrasound features of lymph nodes as input. But cervical lymph nodes are widely distributed (mainly in 6 regions) and there are some limitations in the feature recognition of cervical lymph nodes by ultrasound, especially the lymph nodes in the central area, as well as the special anatomical structures such as posterior trachea, posterior esophagus, retropharyngeal area, and mediastinum, which cannot be displayed well by ultrasound [45]. Meanwhile, researches in modeling, diagnosis, and treatment have confirmed that some ultrasonic features of primary lesions are related to lymph node metastasis [46, 47]. Our experiment also demonstrated that we can better identify lymph node metastasis in different regions through imaging features of primary lesions. This was the reason why no lymph node features were used as input in the present study.

Unlike the analysis of normal cancer [48, 49], lymph node metastasis is detected through postoperative pathology (gold standard) [50]. The inclusion criteria of this study were those who underwent extensive neck lymph node dissection to ensure the accurate diagnosis of LNM. The potential risk of lymph node metastasis has led to many PTC patients receiving total thyroidectomy, lymph node dissection, and other treatments, resulting in widespread overtreatment. Therefore, we hope to build a diagnostic model of preoperative LNM to help realize accurate identification of high-risk patients with LNM in this population to reduce overtreatment.

We constructed five early diagnosis models of LNM by combining the preoperative ultrasound features and ultrasound image features. These models were chosen for the convenience to extract the imaging features of the focus area of PTC. The strategy in construction of the five diagnostic models was different, and finally, we founded that the top three parameters are more important than the others. These results present further evidence for a systematic review and meta-analysis in previous studies, which indicated that patient gender is a factor associated with lymph node metastasis in T1 colorectal cancer [51]. The clinical significance lies in helping the clinicians in early diagnosis, which not only reduces the workload of clinicians but also cut off the suffering of patients [52–54]. The previous studies utilized deep learning algorithms for detection of lymph node metastases, while broad learning algorithms were rarely utilized [54]. Deep learning models spend too much time in the training stage and BLS can greatly reduce the time cost in training the model [53, 54]. This was also the major innovation of our study.

## 4. Conclusion

In this paper, five early diagnostic models were developed from random forest and integrated with the BLS to obtain experimental results with population informatics, clinical data, and ultrasonic characteristics. There was no significant difference between the combining of BLS and random forest and random forest was chosen to make predictions for the model. The most important feature map statistics show the maximum diameter of the nodule. It was the most important variable, followed by the GLSZM zone entropy and hence should be employed in subsequent studies [55–60].

## Figures and Tables

**Figure 1:** (a) Flow chart for the model development and validation. (b) Characteristics of the diagnostic models.

**Figure 2:** ROC curves of the four models in training and testing sets.

**Figure 3:** The ROC curve of Model 4 and Model 5 in training and testing sets.

**Figure 4:** Features importance map.

**Figure 5:** Ultrasonic features AUC: testing set on the left and training set on the right (carcinoembryonic antigen, maximum diameter of nodule, age, GLSZM zone entropy, sex, calcification, aspect ratio, and relative capsule position in turn, which are modified according to translation.

**Table 1:** Sensitivity analysis before and after gap-filling.

Variables	Missing number	Before filling (*n* = 428)	After filling (*n* = 428)	Statistics	*P*
Carcinoembryonic antigen, M(Q_1_,Q_3_)	17 (3.97%)	1.42 (0.88, 2.10)	1.42 (0.89, 2.07)	*Z* = −0.066	0.948
Free triiodothyroxine, mean ± SD	8 (1.87%)	5.15 ± 1.31	5.16 ± 1.32	*t* = −0.06	0.949
Free thyroxine, mean ± SD	8 (1.87%)	18.29 ± 4.76	17.96 ± 3.70	*t* = 1.12	0.261
Thyroid stimulating hormone, M(Q_1_,Q_3_)	8 (1.87%)	1.93 (1.12, 3.17)	1.96 (1.15, 3.19)	*Z* = 0.368	0.713
Thyroid globulin antibody, M(Q_1_,Q_3_)	8 (1.87%)	19.04 (12.98, 66.89)	18.66 (12.97, 57.48)	*Z* = −0.397	0.691
Maximum diameter of nodule, M(Q_1_,Q_3_)	1 (0.23%)	0.80 (0.50, 1.20)	0.80 (0.50, 1.20)	*Z* = −0.055	0.956

**Table 2:** Characteristics comparison for the training and testing sets.

Variables	Total (*n* = 973)	Training set (*n* = 681)	Testing set (*n* = 292)	Statistics	*P*
*Gender, n (%)*					
Male	207 (21.27)	143 (21.00)	64 (21.92)	*χ* ^2^ = 0.103	0.748
Female	766 (78.73)	538 (79.00)	228 (78.08)		

Age, mean ± SD	44.74 ± 11.25	44.66 ± 11.05	44.91 ± 11.70	*t* = −0.32	0.752
BMI, mean ± SD	23.87 ± 3.39	23.90 ± 3.43	23.82 ± 3.29	*t* = 0.30	0.763
Carcinoembryonic antigen, M(Q_1_, Q_3_)	1.34 (0.86, 2.02)	1.34 (0.84, 2.02)	1.33 (0.89, 2.05)	*Z* = 0.067	0.947
The free triiodide, M(Q_1_, Q_3_)	5.10 (4.60, 5.50)	5.10 (4.60, 5.50)	5.00 (4.60, 5.50)	*Z* = −0.201	0.841
Free thyroxine, mean ± SD	18.61 ± 5.03	18.58 ± 4.80	18.67 ± 5.55	*t* = −0.24	0.812
T stimulating hormone, M(Q_1_, Q_3_)	1.91 (1.11, 3.19)	1.94 (1.15, 3.25)	1.78 (1.06, 2.99)	*Z* = −1.374	0.169
T globulin antibody, M(Q_1_, Q_3_)	20.92 (12.98, 78.98)	20.92 (13.04, 83.68)	19.11(12.27, 73.34)	*Z* = −0.982	0.326
*Part, n (%)*					
Ru	105 (10.79)	73 (10.72)	32 (10.96)	*χ* ^2^ = 6.065	0.416
Right middle school	266 (27.34)	199 (29.22)	67 (22.95)		
Lower right	148 (15.21)	101 (14.83)	47 (16.10)		
Left	73 (7.50)	47 (6.90)	26 (8.90)		
Left middle school	237 (24.36)	167 (24.52)	70 (23.97)		
The lower left	100 (10.28)	64 (9.40)	36 (12.33)		
Isthmus	44 (4.52)	30 (4.41)	14 (4.79)		

Max diameter of nodule, M(Q_1_, Q_3_)	0.80 (0.54, 1.20)	0.80(0.53, 1.20)	0.80(0.57, 1.31)	*Z* = 0.867	0.386
*Form, n (%)*					
Rules	95 (9.76)	64 (9.40)	31 (10.62)	*χ* ^2^ = 1.327	0.515
Under-rule	318 (32.68)	217 (31.86)	101 (34.59)		
Irregular	560 (57.55)	400 (58.74)	160 (54.79)		

*Boundary, n (%)*					
Clear	170 (17.47)	113 (16.59)	57 (19.52)	*χ* ^2^ = 1.226	0.542
Lack of clarity	368 (37.82)	261 (38.33)	107 (36.64)		
Unclear or vague	435 (44.71)	307 (45.08)	128 (43.84)		

*Aspect ratio, n (%)*					
≤1	415 (42.65)	282 (41.41)	133 (45.55)	*χ* ^2^ = 1.431	0.232
>1	558 (57.35)	399 (58.59)	159 (54.45)		

*Composition, n (%)*					
Cystic or almost totally cystic	1 (0.10)	1 (0.15)	0 (0.00)	Fisher	1.000
Capsule solidity	19 (1.95)	13 (1.91)	6 (2.05)		
Real or almost all real	953 (97.94)	667 (97.94)	286 (97.95)		

*Echo, n (%)*					
Isoechoic or hyperechoic	5 (0.51)	3 (0.44)	2 (0.68)	Fisher	0.898
Low echo	926 (95.17)	649 (95.30)	277 (94.86)		
Extremely low echo	21 (2.16)	14 (2.06)	7 (2.40)		
Mixed echo	21 (2.16)	15 (2.20)	6 (2.05)		

*Calcification, n (%)*					
No calcification	362 (37.20)	262 (38.47)	100 (34.25)	Fisher	0.293
Coarse calcification	62 (6.37)	47 (6.90)	15 (5.14)		
Eggshell calcification	6 (0.62)	5 (0.73)	1 (0.34)		
Microcalcification	543 (55.81)	367 (53.89)	176 (60.27)		

*Relative coating position, n (%)*					
Stay away from	398 (40.90)	286 (42.00)	112 (38.36)	*χ* ^2^ = 1.123	0.570
Cling	485 (49.85)	333 (48.90)	152 (52.05)		
Breakthrough	90 (9.25)	62 (9.10)	28 (9.59)		

TI_DS classification, *n* (%)				*χ* ^2^ = 0.812	0.937
*LNM transfer, n (%)*					
No	576 (59.20)	410 (60.21)	166 (56.85)	*χ* ^2^ = 0.953	0.329
Yes	397 (40.80)	271 (39.79)	126 (43.15)		

T: thyroid; TI_DS: ultrasonic thyroid imaging and data system; LNM: lymph node metastases.

**Table 3:** The predictive performance of these models in the training and testing sets.

Models	Cut-off	Sensitivity (95% CI)	Specificity (95% CI)	PPV (95% CI)	NPV (95% CI)	AUC (95% CI)	Accuracy (95% CI)
Model 1^a^	0.348	0.849 (0.806–0.891)	0.851 (0.817–0.886)	0.790 (0.744–0.837)	0.895 (0.864–0.925)	0.913 (0.893–0.934)	0.850 (0.823–0.877)
Model 1^b^	0.348	0.738 (0.661–0.815)	0.771 (0.707–0.835)	0.710 (0.632–0.788)	0.795 (0.733–0.857)	0.813 (0.762–0.863)	0.757 (0.708–0.806)
Model 2^a^	0.437	0.808 (0.761–0.855)	0.868 (0.836–0.901)	0.802 (0.755–0.849)	0.873 (0.840–0.905)	0.913 (0.892–0.934)	0.844 (0.817–0.872)
Model 2^b^	0.437	0.730 (0.653–0.808)	0.789 (0.727–0.851)	0.724 (0.647–0.802)	0.794 (0.732–0.856)	0.818 (0.769–0.868)	0.764 (0.715–0.812)
Model 3^a^	0.360	0.886 (0.848–0.924)	0.827 (0.790–0.863)	0.772 (0.725–0.818)	0.916 (0.888–0.944)	0.941 (0.925–0.957)	0.850 (0.823–0.877)
Model 3^b^	0.360	0.762 (0.688–0.836)	0.723 (0.655–0.791)	0.676 (0.599–0.753)	0.800 (0.736–0.864)	0.821 (0.772–0.871)	0.740 (0.689–0.790)
Model 4^a^	0.500	0.823 (0.777–0.868)	0.966 (0.948–0.983)	0.941 (0.911–0.971)	0.892 (0.863–0.921)	0.984 (0.977–0.990)	0.909 (0.887–0.931)
Model 4^b^	0.500	0.667 (0.584–0.749)	0.910 (0.866–0.953)	0.848 (0.778–0.919)	0.782 (0.724–0.841)	0.857 (0.811–0.902)	0.805 (0.759–0.850)

^a^Using the training set; ^b^using the testing set. PPV: positive predictive value; NPV: predictive value; AUC: area under the curve; CI: confidence internal.

**Table 4:** The predictive performance of lymph node metastasis by BLS feature learning.

Models	Cut-off	Sensitivity (95% CI)	Specificity (95% CI)	PPV (95% CI)	NPV (95% CI)	AUC (95% CI)	Accuracy (95% CI)
Model 4^a^	0.500	0.823 (0.777–0.868)	0.966 (0.948–0.983)	0.941 (0.911–0.971)	0.892 (0.863–0.921)	0.984 (0.977–0.990)	0.909 (0.887–0.931)
Model 4^b^	0.500	0.667 (0.584–0.749)	0.910 (0.866–0.953)	0.848 (0.778–0.919)	0.782 (0.724–0.841)	0.857 (0.811–0.902)	0.805 (0.759–0.850)
Model 5^a^	0.465	0.959 (0.936–0.983)	0.973 (0.958–0.989)	0.959 (0.936–0.983)	0.973 (0.958–0.989)	0.995 (0.992–0.998)	0.968 (0.954–0.981)
Model 5^b^	0.465	0.778 (0.705–0.850)	0.843 (0.788–0.899)	0.790 (0.719–0.862)	0.833 (0.777–0.890)	0.853 (0.806–0.901)	0.815 (0.771–0.860)

^a^Using the training set; ^b^using the testing set. PPV: positive predictive value; NPV: predictive value; AUC: area under the curve; CI: confidence internal.

## Data Availability

All the data to support the experiments and findings in this study are available from the corresponding authors upon request.
